# Sensor potency of the moonlighting enzyme-decorated cytoskeleton: the cytoskeleton as a metabolic sensor

**DOI:** 10.1186/1471-2091-14-3

**Published:** 2013-02-11

**Authors:** Vic Norris, Patrick Amar, Guillaume Legent, Camille Ripoll, Michel Thellier, Judit Ovádi

**Affiliations:** 1 EA 3829, Faculté des Sciences de l’Université de Rouen, 76821, Mont Saint Aignan Cedex, France; 2 DYCOEC, CNRS (GDR 2984), CORIA, Université de Rouen, Rouen, France; 3 LRI, Univ. Paris Sud, CNRS, UMR 8623, & INRIA Saclay, F-91405, Orsay, Cedex, France; 4 Institute of Enzymology, Research Center for Natural Sciences, Hungarian Academy of Sciences, Budapest, Hungary

## Abstract

**Background:**

There is extensive evidence for the interaction of metabolic enzymes with the eukaryotic cytoskeleton. The significance of these interactions is far from clear.

**Presentation of the hypothesis:**

In the cytoskeletal integrative sensor hypothesis presented here, the cytoskeleton senses and integrates the general metabolic activity of the cell. This activity depends on the binding to the cytoskeleton of enzymes and, depending on the nature of the enzyme, this binding may occur if the enzyme is either active or inactive but not both. This enzyme-binding is further proposed to stabilize microtubules and microfilaments and to alter rates of GTP and ATP hydrolysis and their levels.

**Testing the hypothesis:**

Evidence consistent with the cytoskeletal integrative sensor hypothesis is presented in the case of glycolysis. Several testable predictions are made. There should be a relationship between post-translational modifications of tubulin and of actin and their interaction with metabolic enzymes. Different conditions of cytoskeletal dynamics and enzyme-cytoskeleton binding should reveal significant differences in local and perhaps global levels and ratios of ATP and GTP. The different functions of moonlighting enzymes should depend on cytoskeletal binding.

**Implications of the hypothesis:**

The physical and chemical effects arising from metabolic sensing by the cytoskeleton would have major consequences on cell shape, dynamics and cell cycle progression. The hypothesis provides a framework that helps the significance of the enzyme-decorated cytoskeleton be determined.

## Background

The eukaryotic cytoskeleton is a system of protein filaments within the cell that confers structural integrity, exerts force, responds to stimuli, drives the cell cycle, performs mechanotransduction and produces motion. Structural integrity results from the cytoskeleton being a robust meshwork extending throughout the cytoplasm. Responses to stimuli result from the cytoskeleton being a highly dynamic structure, in which filaments associate with or dissociate from one another, slide, grow and shrink, and provide tracks for motor proteins and their cargoes. Changes in cell shape and volume result from interaction of the cytoskeleton with membrane-bound receptors, which include growth factor receptors.

A large and growing body of evidence also attests to the interaction of the cytoskeleton with a variety of metabolic enzymes [1] and references therein. It has been argued that the fundamental problem that confronts all cells is that of generating reproducible phenotypes on which natural selection can act [2]. Clearly, cells face the enormous challenge of generating a small set of phenotypes – that must be coherent with the myriads of internal and external conditions – from hundreds of thousands (if not millions) of different constituents. Ensuring this coherence entails sensing and integrating a wide diversity of chemical and physical information so as to converge onto a few outputs. These outputs must affect many of the systems and hence must be extremely well-connected. Just how cells achieve this is far from clear.

One evident possibility is that metabolism and signaling are tightly linked to the ultrastructure and dynamics of the cytoskeleton. The concept of “functioning-dependent structure” (FDS) was developed to describe either those structures that only form when their constituents are performing a task (and that disappear when that these constituents cease performing the task) or the inverse, namely those structures that only form when the constituents are *not* performing their task [3]. A metabolic FDS comprises enzymes (often sequential in a pathway) that, for example, assemble into the higher order structure only when these enzymes are catalyzing their reactions; in the absence of substrate these enzymes are therefore free [4]. Modeling the behavior of such enzymes has revealed that they may be able to generate waves of metabolites and hence play a role in signaling [5]. A related concept is that of “ambiquitous” enzymes which can occupy two different positions in the cell, for example, free or associated with the cytoskeleton [6]. The concept of ambiquity itself is related to that of ‘moonlighting’, in which a protein has multiple, independent functions and plays more than one role in an organism, however, these functions do not arise from gene fusions, splice variants, or post-translational modifications [7]. Such moonlighting often involves the dynamic, multi-functional cytoskeleton, which is therefore well placed to transduce a wide variety of internal and external signals.

Under strong evolutionary pressures, bacteria, which are highly structured, have had the time and the numbers to find the solutions to many problems. One of these solutions is metabolic sensing. In *Bacillus subtilis*, for example, the association of the glucosyltransferase, UgtP, with the tubulin-like FtsZ couples cell division to nutrient availability [8]. Here we use the concepts of FDS, ambiquity and moonlighting to explore the possibility that metabolism and signaling are linked via enzyme associations with the cytoskeleton. We propose that a functioning-dependent co-assembly of metabolic enzymes plus cytoskeleton – a type of *enzoskeleton*[9] – could integrate metabolic information and thereby help solve the problem of generating a coherent phenotype.

## Presentation of the hypothesis

### Sensing at what level?

It might be argued that sensing is done by individual proteins (or other macromolecules) rather than by macromolecular assemblies *alias hyperstructures*[10]. It might even be argued that sensing is done by individual amino acids within proteins. Although all these levels of organization are involved, the crux of the matter is which level provides the most meaningful explanation for the event of interest? Lemke has suggested that each new emergent level of organization in the dynamics of a complex self-organizing system functions to re-organize variety on the level below as meaning for the level above [11]. In the 3-level paradigm of Salthe, units on level N (e.g. the tubulin cytoskeleton) are constituted by interactions among the units at the lower level (N-1) (e.g. tubulin and enzymes), but that of all the possible configurations which such interactions might produce at level N, only those actually occur which are allowed by boundary conditions set at level (N+1) (e.g. the cell itself) [12]. We have adopted this sort of thinking in proposing that the existence of hyperstructures, at a level intermediate between the macromolecule and the cell, allows cells to reduce background noise from the lower level of macromolecules and hence facilitate the emergence of a coherent pattern at the higher level of the cell itself, thus producing the desired phenotype [10]. If then, we are to understand the response of the cell to metabolic information, it should be at the level of intracellular assemblies or hyperstructures. A good example of this is the proposal that the amplification of the signal in bacterial chemotaxis depends on the size of the chemotactic array or hyperstructure [13]. In this context, it has also been argued that for systems at different levels of biological organization: “three general features can be discerned: (1) a high off-rate that allows energy-dependent exploration of an assembly landscape, and selection of a functional steady state; (2) two- or multi-statedness of the components of the system; and (3) induced collapse of the whole system into singular states” [14]. The dynamical cytoskeleton has therefore the right characteristics to exploit (sense) the information in enzymes, much as a company exploits the information in the registered letters carried by postmen.

### The cytoskeletal integrative sensor hypothesis

The binding to microtubules and to actin filaments of enzymes responsible for catalyzing different metabolic pathways allows the cytoskeleton to sense and integrate metabolic activity (Figure 1). This sensing and integration occur via alterations in the physical stability and dynamics of cytoskeletal filaments, in the rates of hydrolysis of GTP and ATP by cytoskeletal elements and associated enzymes, and in the levels of metabolites. The consequence of this integration at both cellular and tissue levels is a regulation that determines the efficiency of pathways, the moonlighting functions of enzymes, and the coherence of the phenotype.

**Figure 1:** **Simple schema of metabolite-sensing.** (**A**) The dynamic equilibrium between the polymeric forms of a cytoskeletal protein (red rectangles) depends on some enzymes (green pentagons and brown circles) binding and stabilizing the polymers when these enzymes are either active in catalyzing their cognate reactions (presence of star) or when these enzymes are inactive (absence of star). Only one type of cytoskeletal protein is shown. (**B**) The web of interactions involved in sensing changes in levels of metabolites by the cytoskeleton. The red arrows inside the ellipse represent the equilibrium between the polymeric forms that is at the heart of the sensing. The blue arrows represent the flow of information through the network following a change in metabolite levels. The thick blue arrow represents initial effects of changes in metabolite levels on the equilibrium between cytoskeletal structures with and without associated enzymes. Thin blue arrows represent subsequent effects on cytoskeletal dynamics, enzyme activation, enzyme-enzyme association and on ATP/GTP levels.

### The mechanism

The organization of the cytoskeleton is affected by specific proteins such as Microtubule-Associated Proteins or MAPs. In neurons, for example, MAPs bind strongly to MTs to make them relatively stable (in the sense that they can be isolated) whilst in higher plant cells, MAPs play a major role in the various dynamic transformations undergone by the MT network [15]. The cytoskeleton also binds less strongly to certain enzymes and the association is transient, allowing the cytoskeleton to remain dynamic. Association with the cytoskeleton requires specific conformers of enzymes, thus the cytoskeleton binds some enzymes when they are active, that is, catalyzing their reactions, whilst it binds others when they are inactive. The entire cytoskeletal hyperstructure with its associated enzymes is therefore an FDS that can act as a sensitive intracellular sensor.

The levels of nucleotides such as ATP and GTP affect the binding by the cytoskeleton of enzymes; reciprocally, the ultrastructure of the cytoskeleton affects the rate and extent of the hydrolysis of these nucleotides as catalyzed by either the cytoskeleton itself and/or the cytoskeleton-associated enzymes.

Since the cytoskeleton and GTP and ATP are central players in cell architecture and in related physiological functions, stabilization of the cytoskeleton and regulation of nucleotide levels then allow the enzyme-associated cytoskeleton to act as a sensor that helps determine the phenotype of the cell.

### The evidence

Macromolecular interactions, compartmentation, channeling and ambiquity have a long history (for references see [16]). It now turns out that over a hundred proteins, including many involved in metabolism, change their distribution in the yeast, *Saccharomyces cerevisiae*, in response to altered metabolic conditions, moreover, association and dissociation of enzyme foci can be controlled by availability of specific metabolites, leading to the suggestion that metabolite-specific, reversible protein assemblies are common [17,18]. Some of the proteins involved may interact with the cytoskeleton (for example, those involved in purine synthesis, see below) opening up the possibility that the dynamics of these enzyme hyperstructures is coupled to the dynamics of the cytoskeleton. The actin cytoskeleton in *S*. *cerevisiae* also undergoes a major change as cells go from a quiescent state to growth. In the quiescent state, actin is in the form of immobile bodies; on resumption of metabolic activity following refeeding, actin again forms a dynamic network [19]. The tubulin cytoskeleton in oligodendrocytes undergoes a major change as they extend filopodial processes and contact axons, prior to myelin ensheathment; during this development, oligodendrocytes are metabolically the most active cells in the CNS [20]. This unique change, rearrangement of the microtubules during differentiation, is associated with the MT cytoskeleton binding to specific (marker) proteins such as myelin basic protein and TPPP/p25 [21].

### Binding of cytoskeleton to enzymes involved in energy metabolism

An extensive body of literature attests to the interactions of metabolic enzymes with microfilaments of actin and with microtubules. Interactions with microtubular proteins have been observed for the glycolytic kinases, hexokinase (HK), phosphofructokinase (PFK) and pyruvate kinase (PK) as well as aldolase (for references see [22]). These interactions between tubulin and metabolic enzymes lead to the formation of distinct hyperstructures (Figure one in [22]). MT bundling results from the binding of MTs to glyceraldehyde-3-phosphate dehydrogenase (GAPDH). MTs also interact with a wide variety of enzymes, including translation factors, RNA-binding proteins, signaling proteins and metabolic enzymes [23]. Interactions between MTs and enzymes extend to interactions between MTs and enzyme hyperstructures, as suggested by evidence that the MT network determines the distribution and activity of purinosomes in which purine is synthesized in HeLa cells [24] (but see [25]). In the case of actin, interaction of microfilaments with glycolytic enzymes led, in the case of studies on muscle, to the conclusion that, in general, “actin binds enzymes”. Even filamentous actin from yeast binds enzymes, albeit more weakly, and such microfilaments bind aldolase and GAPDH [26,27]. For example, actin bundling and the formation of actin-based hyperstructures results from interaction with aldolase in XTH-2 cells from *Xenopus laevis* and keratocytes [28]. In plants, protein–protein interactions have been found between actin and enzymes that include cytosolic aldolase, three GAPDH isoforms and two enolase isoforms, as well as between tubulin and enzymes that include aldolase, GAPDH and sucrose synthase [29].

Interactions between MTs and enzymes can be extended to interactions between MT motor proteins and docking proteins that connect the motor proteins to their cargoes. Identification of the docking proteins has shown that they are often moonlighting and have other functions in, for example, signaling and metabolism (for references see [30]). These interactions include those: between a kinesin-related protein, rabkinesin-6, and a small GTPase, Rab6, involved in membrane trafficking; between a dynactin complex and spectrin, which binds to lipids and connects membrane proteins with actin filaments; between dynein and glucose-6-phosphate dehydrogenase [31].

Finally, dynamic interactions between microfilaments and MTs, which have been proposed to play a major role in neuronal growth cones [32], have recently been described in the model plant, *Arabidopsis thaliana*[33]. We cannot exclude the possibility that such interactions involve metabolic enzymes thereby taking cytoskeletal sensing to a very high level of integration. Some support for this possibility is given by the findings that (1) a fraction from tobacco pollen tubes containing PFK, homocysteine methyltransferase, pyruvate decarboxylase, and glucan protein synthase promoted the bundling of actin microfilaments and the interaction of these microfilaments with microtubules [34] and (2) in apple pollen, the binding of actin filaments to a transglutaminase (which catalyses the reaction between acyl acceptor glutamyl residues and amine donors) led to the aggregation of actin and to a similar aggregation using tubulin [35]. That said, the binding of metabolic enzymes to both microfilaments and MTs at the same time may be rare given that the binding of enzymes to the different cytoskeletal filaments is frequently isoform-specific and can vary with the activity state of the enzyme. This is the case of PFK: brain PFK does not bind MTs whilst muscle PFK is relatively inactive when bound to MTs but fully active when bound to microfilaments [36].

### Functioning-dependent binding of enzymes to the cytoskeleton

The essence of our interpretation of the following results is that if the binding by the cytoskeleton of an enzyme increases the probability of catalysis (via for example its affinity for its substrate), reciprocally, the cytoskeleton might well have a higher probability of associating with an enzyme that is active in catalysis. In other words, if being bound to a cytoskeletal filament confers a conformation on an enzyme that allows it to bind its substrate then the activation of the free enzyme by substrate might promote the binding to this enzyme to the filament.

Microtubule binding to glycolytic enzymes alters the catalytic and regulatory properties of these enzymes (see Table one in [22]). Such binding increases HK activity (resulting in enhanced glycolytic flux in brain tissue) but this does not influence MT dynamics and structure. MT binding to PFK, which is direct [37], leads to a periodic cross-linking of the MTs and decreases enzyme activity (by inducing dissociation of the tetrameric enzyme). MT binding to PK does not affect its activity but impedes MT assembly. The binding by MTs of the individual enzymes is influenced by enzyme-enzyme interactions. Formation of an aldolase-PFK complex prevents the association of PFK with MT or, put differently, results in PFK’s detachment from the MT. Within this complex, PFK is stable and maintains its catalytic activity, the allosteric property is, however, abolished [22].

Results on the interaction of microfilaments with PFK, GAPDH and aldolase can also be interpreted as consistent with such interaction depending on the state of the enzyme. Binding to filamentous actin is known to activate PFK. Recently, it has been shown that insulin signaling increases the association of PFK with actin filaments and it was suggested that this association plays a role in the stimulation of glycolysis by insulin [38]. In serum-depleted cells, the cytoplasmic GAPDH is colocalised with actin stress fibers whereas in the presence of serum, this enzyme is distributed homogeneously [26]. In quiescent cells, aldolase is colocalised along stress fibers whereas in motile cells it is behind the ruffles at the leading edge of the cell [39]. In the presence of fructose-1,6-bisphosphate, a G-actin-aldolase mixture polymerizes to a higher viscosity and forms stiffer filaments than pure actin of the same concentration whilst in permeabilized cells in the presence of fructose-1,6-bisphosphate, aldolase goes from association with actin fibers to association with intermediate filaments [28]. In maize, the presence of sucrose is required for the association of sucrose synthase with microfilaments *in vitro* and probably *in vivo*[40].

Interactions between metabolites and the cytoskeleton are closely related to those between enzymes and the cytoskeleton and, in terms of metabolic sensing, are even more direct. It has been found, for example, that cardiac steroids acting via the Na^+^/K^+^-ATPase and the ERK1/2 signaling pathway induce formation of clusters containing not only glycogen synthase and distorted MTs but also glycogen [41].

### Cytoskeletal control of and by ATP/GTP levels

Energy dissipation is critical for the dynamic non-equilibrium behavior of microfilaments and microtubules as when ATP and GTP associated with actin monomers and tubulin dimers, respectively, are irreversibly hydrolyzed into ADP and GDP [42]. How might this be linked to the cytoskeleton sensing metabolic activity? There is ample evidence that the association between cytoskeletal filaments and metabolic enzymes can affect the structural and functional features of both partners in a two-way relationship with nucleoside triphosphate levels; on one hand, the altered hydrolytic potency of the cytoskeletal filaments modifies the nucleoside triphosphate levels, and, on the other hand, the stability, dynamic and hydrolytic activity of the cytoskeleton is modified by the nucleoside triphosphate levels. One example of how GTP or ATP availability affects cytoskeletal dynamics is treadmilling, a nucleoside triphosphate-dependent process in which filament length remains approximately constant while subunits are added to the (+) end and removed from the (−) end of the filaments. The efficiency of MT treadmilling is related to whether tubulin dimers are incorporated into the microtubule treadmill, a process that varies with GTP concentration [43] A second example is the dependence of MT dynamics on MT motor proteins (like Kin-I kinesins), which use ATP hydrolysis to do mechanical work [44]. A third example is the possible control by the GTP level of the polarization of the actin cytoskeleton of migrating cells via small GTPases of the Rho family [45]; in this control, these GTPases are active when bound to GTP and inactive when bound to GDP; this binding is regulated by Guanine Exchange Factors and the opposing GTPase Activating Proteins such that the ratio of binding of GTP versus GDP to the small GTPases reflects the cytosolic level of GTP:GDP and the local concentration of the exchange factors and activating proteins [46]. Actin stress fibers assemble in response to a signaling cascade in which the GTP-bound form of RhoA [47] (1) activates Rho-associated kinase which inhibits the depolymerization of actin filaments (via LIM kinase and actin depolymerizing factor/cofilins) [48], (2) induces contractility (via myosin light chains) [49] and (3) activates formins, Rho-GTPase effector proteins, involved in actin polymerization [50].

What then of the inverse – is there evidence that cytoskeletal dynamics affects the levels of the nucleoside triphosphates? It has been suspected that the dynamics of actin are implicated in the regulation of ATP levels [51] and that MT dynamics affect GTP levels (which in turn might affect those dynamics) [52]. Recently, it has been pointed out that the 10-fold decrease in the GTP/GMP ratio observed in yeast following nutrient changes: “highlights the sensitivity of this ratio (as an) indicator of metabolic status” [53] – and GTP hydrolysis is tightly coupled to the dynamics of polymerization of tubulin subunits [54], a hydrolysis stimulated by MAPs which increases the efficiency of nucleation [55]. (Note that this relationship with MAPs is, again, two-way as shown when GTP impedes the association of the MAP TPPP/p25 with the MT mitotic spindle to arrest mitosis in *Drosophila*[56]).

### Functional consequences of cytoskeletal sensing

There is abundant evidence that, in addition to the metabolic enzymes, other proteins binding to the actin and tubulin cytoskeletons alter their dynamics. In the case of actin, the unregulated polymerization of actin filaments is inhibited in cells by actin monomer-binding proteins such as profilin and Tbeta4 [57]. Nucleators of actin polymerization include the Arp2/3 complex and its large family of nucleation-promoting factors (NPFs), formins, Spire, Cobl, VopL/VopF, TARP and Lmod. These proteins control the time and location for polymerization and influence the structures of the actin networks. Coronin, an important protein in actin dynamics, changes its activity depending on the nucleotidic state of actin [58]. IQGAPs are actin-binding proteins that transmit extracellular signals to the actin network so as to influence mitogenic, morphological and migratory cell behavior [59,60]. In growth cones, ezrin/radixin/moesin (ERM) proteins tether actin filaments to the cell membrane and transmit Nerve growth factor and neurotrophin-3 signals to the actin network, which leads to its remodeling and to the redistribution of adhesion receptors [61]; similarly, the vascular endothelial growth factor receptor 2 transduces the VEGF signal into major actin rearrangements [62]. In *A*. *thaliana*, hexokinase1 interacts with actin; given that a normal functioning actin cytoskeleton is required for hexokinase1 to play its role in glucose signaling, it has been suggested that this enzyme “might alter F-actin dynamics and thereby influence the formation and/or stabilization of cytoskeleton-bound polysomes” [63,64].

It was proposed in 1951 that the cytoskeleton might serve as a cellular ‘nervous system’ [65]. More recently, it has been argued in the case of tubulin that phosphorylation in neuronal MT networks could play the central role in the signaling and encoding required in memory [66]. In line with this, microtubule-associated proteins, such as tau and TPPP/p25, promote MT assembly and stabilize MT networks with phosphorylation regulating these functions [67,68]. Changes in the phosphorylation of tau are correlated with changes in the association of tau with the MT network [69]. Distinct superstructures of the MT network have different binding potencies for metabolic enzymes and motor proteins; this results in altered sensing. A related – extreme – example of this is the hyperphosphorylation of tau which leads to the aggregation of filamentous tau, the consequent activation of axonal protein protein phosphatase 1 and glycogen synthase kinase 3, and the inhibition of axonal transport [70], a critical factor in neurodegenerative diseases [71]. The aggregation of tau may be a protective mechanism that helps avoid the interaction of abnormal tau with the MT network, an interaction that in our hypothesis should result in a major perturbation of MT signaling and its consequences [72], given that the neurofibrillar tangles of tau alter MT dynamics significantly. In many plants, the directional deposition of cellulose microfibrils determines anisotropic growth and cell shape. These microfibrils are made by plasma membrane-located cellulose synthase complexes that are aligned with and that move along cortical microtubules. Since defects in the mobility of these complexes affects the MT network, it has been proposed that “some form of signaling process communicates the cellulose synthesis impairment to microtubules … a direct feedback loop between these complexes and microtubules could be involved” [73]. It is therefore conceivable that this loop includes an effect of the activity of the cellulose synthase complexes on MT binding and dynamics.

There are intriguing relationships between growth factor receptors, cytoskeletal organization, changes in cell shape, the glycolytic flux and the onset of S-phase. Shape changes are central to the cell cycle, which entails major reorganizations of both microfilaments and MTs. In the case of microfilaments, it should be noted that some actin exists in the form of a perinuclear actin cap and associated focal adhesions that shape the nucleus during interphase and that mediate mechanotransduction, motility, polarization and differentiation [74]. External signal molecules, such as growth factors and extracellular matrix components, act via signal transduction pathways (which include those based on MAP kinase and PI-3 kinase) to determine whether the cell in G1 phase continues proliferation or undergoes apoptosis, differentiation, or quiescence. Actin dynamics have been proposed as important in this progression through G1 given actin’s role in these pathways, in transcription (see below) and in cell shape and structure [75]. Both glutamine and glucose are needed for progression from G1 into S phase. This progression is inhibited by inactivation of a critical enzyme in glutaminolysis, glutaminase 1, or by inactivation of the glycolysis-promoting enzyme, 6-phosphofructo-2-kinase/fructose-2,6-bisphosphatase isoform 3 [76]. Signal transduction pathways, for example, involving molecular chaperones and immunophilins, also influence MT dynamics to determine cell cycle progress and differentiation [72].

An important consequence of cytoskeletal sensing is on transcription. When the F-actin:G-actin levels are low, G-actin binds to MAL and prevents MAL activating the SRF transcription factor whilst when the F-actin:G-actin levels are high, MAL is free to activate SRF. This has led to the question being raised as to whether “altered F-actin:G-actin ratios arising during guidance responses mediated by UNC-115/ablim or other cytoskeletal regulators in the growth cone influence gene expression during guidance” [32].

Where do isoforms fit in? In the integrative sensing hypothesis, cytoskeletal binding to different isoforms should have different functional consequences. MTs bind PK, an isoform of which, pyruvate kinase M2, is a major regulator of the glycolytic flux in tumor cells; this has led to the suggestion that M2-PK is a metabolic sensor which regulates cell proliferation, cell growth and apoptotic cell death in a glucose supply-dependent manner [77]. Enolase is a glycolytic enzyme acting on 2-phosphoglycerate and, in higher vertebrates, exists as cell-type specific α and/or β isoforms. MTs interact with both isoforms, and the direct binding of tubulin to enolase is abolished by its substrate [78]. During myogenic differentiation, the level of the β subunit increased and became partially aligned along the MT network. At various stages of this differentiation, MTs were decorated by the different enolase isoforms depending on the dynamic state of the MTs and the abundance of the isoforms [78]. The fact that the changes in the MT dynamics, which accompany the transition from myoblast to myotubes, may be related to the 2-phosphoglycerate level and to isoform abundances would be consistent with the MT network acting as a sensor to control this transition. In this context of relationships between MT structures, binding and function, an interesting variant is the binding of the anti-cancer agent KAR2 by mitotic spindle MTs but not by interphase MTs which has the functional consequence of inhibiting cell division [79].

## Testing the hypothesis

The following predictions and corollaries (in the case of isoforms) of the hypothesis could readily be tested experimentally or by simulation and modeling:

1/ *Isoform differences*. The numerous isoforms of actin and tubulin occurring within the same cell should differ in their capacity to bind enzymes and, reciprocally, the isoforms of enzymes should differ in their affinities for microfilaments and microtubules. Some *in vitro* evidence exists already for this insofar as the dissociated form of the M (muscle) isoform of PFK binds to MT but the C (brain) isoform, which is a stable tetramer, does not [80].

2/ *Metabolism to cytoskeletal dynamics and back to metabolism*. The state of the metabolism should influence, *via* post-translational modifications to the cytoskeleton-binding enzymes and to actin and tubulin themselves, the nature of the cytoskeleton so as to determine the binding and activity of enzymes; reciprocally, this binding should then determine metabolic activity. The prediction is that there would be a relationship between alterations to the sites on tubulin and actin that undergo post-translational modification and cytoskeletal interaction with metabolic enzymes.

3/ *Cytoskeletal dynamics and ATP*/*GTP levels*. The changes in efficiency of ATP and GTP hydrolysis that result from the changes in the ultrastructure of the cytoskeleton (as described in 1/ and 2/) should be sufficient to cause changes in metabolism and signaling that affect the phenotype. Measurement (and simulation, see 4/ below) of the intracellular levels of ATP and GTP under different conditions of cytoskeletal dynamics and enzyme-cytoskeleton binding should reveal whether this is sufficient to significantly affect local and perhaps global levels and ratios of ATP and GTP and related nucleotides. In some cases, it is conceivable that changes in the level and ratios of nucleotides might be masked by, for instance, an up-regulation of the activity of mitochondria (which could itself be tested for).

4/ *Signaling gradients*. Non-homogeneous spatio-temporal distributions of metabolites with a potential for signaling (as well as the distribution of the enzymes themselves) should be generated by functioning-dependent association or disassociation of enzymes from cytoskeletal filaments. Such distributions could be revealed by simulation with stochastic automata such as HSIM [81] which has been used to show that confining metabolic enzymes to a hyperstructure can generate a spatial gradient of the product. They might even be revealed by using a combination of isotope-labeled molecules such as ^13^C-glycogen and Secondary Ion Mass Spectrometry [82].

5/ *Cytoskeletal relationships with moonlighters*. Moonlighting enzymes [83,84] should often have a special relationship with the cytoskeleton with, for example, their multiple functions being related to their being bound to, or separate from, the cytoskeleton. Changes in the levels of glyceraldehyde-3-phosphate and of D-glycerate 1,3-bisphosphate – and hence changes in growth rates and even metastatic potential – might be expected to result from modifications to GAPDH that increase or decrease its affinity for microtubules (and/or microfilaments) and from modifications to microtubules and microfilaments (e.g. via drugs) that affect the binding of GAPDH to the cytoskeleton. Such changes in the level of the enzymes would have to be distinguished from those resulting simply from secondary changes to the catalytic activity of the enzymes.

6/ *Gene expression*. In the case of isoforms, gene expression is clearly involved during myoblast differentiation, when cytoskeletal reorganization and, in particular, the regulation of microtubule dynamics, lead to sarcomere formation (see above). This complex process requires ATP, which is supplied by glycolysis, and the association of different isoforms of enolase to the microtubule system [78]; significantly, the fusion of myoblast microtubules leading to myotube formation is coupled with a large increase in the expression of β enolase [85]. In the case of moonlighting enzymes, coherent effects on the patterns of gene expression should result from changes to the cytoskeletal binding of, for example, GAPDH, given that this enzyme is part of the *OCAS* transcriptional coactivator complex [86].

7/ *Cell shape*, *volume and the cell cycle*. Alterations to metabolic enzymes (or to growth factor receptors) that result in their adopting either an active conformation in the presence of substrate or an inactive conformation in the presence of substrate should alter cytoskeletal dynamics so as to advance or retard, respectively, the onset of S-phase. Such alterations should also affect shape and volume, consistent with a cytoskeleton-mediated sensing of metabolism.

## Implications of the hypothesis

The cytoskeletal integrative sensor hypothesis is an attempt to answer the question of how cells sense and integrate a wide diversity of chemical and physical information so as to converge onto a few outputs and generate a coherent phenotype. This hypothesis is in itself insufficient but it can be combined with other, complementary, hypotheses to give an integrated picture of cell functioning.

One of these hypotheses is based on the possibility of ion condensation on the cytoskeleton [87]. Positive counterions such as potassium, magnesium, calcium and polyamines can condense onto negatively charged linear polymers [88]. Such condensation leads to the counterions being delocalized and diffusing in the near region in intimate contact with the polymer or other surface [89]. Condensation occurs at a critical value of the charge density of the polymer and resembles a phase transition in that it occurs in an abrupt fashion (for references see [87]). Since the activity of protein kinases and phosphatases can be modulated by ions, condensed ions on protein filaments might play a major role in the phosphorylation/dephosphorylation of a wide variety of protein filaments by filament-associated kinases/phosphatases. In this hypothesis, calcium condensation/decondensation on the macromolecular network creates coherent patterns of protein phosphorylation that transduce signals [87]. One of the attractive features of this hypothesis is that changes in temperature and in the tensional state of the macromolecular network cause changes in ion condensation on this network hence allowing it to integrate chemical and physical signals. Divalent ion condensation can also occur in vitro on MTs or actin microfilaments [90-94]. Since both actin and tubulin are negatively charged, the possibility exists that ion condensation on MTs and microfilaments occurs in vivo, as discussed in the case of the bacterial tubulin, FtsZ [95]. In the case of magnesium, condensation of this ion could provide a powerful basis for the activation of enzymes associated with the cytoskeleton whilst decondensation could activate enzymes free in the cytoplasm. Note too that cytoskeleton-associated enzymes could undergo conformational changes due to mechano-transduction by the cytoskeleton [96,97] and that such changes can modulate catalysis [98]; this relationship may be two-way.

A second relevant, integrative hypothesis involves the mechano-transduction properties of the cytoskeleton and associated structures such as focal adhesion complexes [99,100] which contain signaling proteins like Focal Adhesion Kinase, G-proteins like RhoA and stretch-sensitive proteins like ion channels and Talin. The nature of the extracellular matrix affects the composition, structure and size of focal adhesions. Focal adhesions help determine the state of the attached cytoskeleton which, in our proposal, affects metabolism. In this way, classical mechano-transduction signaling pathways could be integrated with metabolism at the level of the cytoskeleton.

A third integrative hypothesis of relevance is that of the cell as being a set of functioning-dependent hyperstructures in which, first, the functioning of an enzyme determines whether or not that enzyme binds to related enzymes and, second, enzymes that are free (i.e. unbound) are degraded preferentially [101]. There is therefore spatial or configurational control over phenotype. These ideas are compatible with the integrative sensing hypothesis insofar as the actin and tubulin cytoskeletons plus their associated enzymes might constitute ‘first among equals’ in the class of functioning-dependent hyperstructures. For example, an enzyme activated by substrate could bind to the cytoskeleton where it would be safe from proteases. There are echoes here of molecular complementarity whereby, first, the binding of biomolecules to one another often alters their physiological activities, and conversely, molecules with closely related physiological activities often bind to one other, and second, the binding of compounds to one another protects them and leads to their accumulation [102,103]. Finally, in the cytoskeletal sensing hypothesis, the activity of numerous enzymes may be transduced by cytoskeletal dynamics into levels of ATP and GTP, two simple outputs with myriad connections to cellular processes.

## Abbreviations

MT: Microtubule; FDS: Functioning-dependent structure; PFK: Phosphofructokinase; GAPDH: Glyceraldehyde-3-phosphate dehydrogenase; TPPP: Tau and tubulin polymerization-promoting protein.

## Authors’ contributions

All authors contributed equally to the ideas and to the writing of the manuscript. All authors read and approved the final manuscript.
